# The Role of Intelligence in Posttraumatic Stress Disorder: Does it Vary by Trauma Severity?

**DOI:** 10.1371/journal.pone.0065391

**Published:** 2013-06-10

**Authors:** Naomi Breslau, Qiaoling Chen, Zhehui Luo

**Affiliations:** Department of Epidemiology and Biostatistics, College of Human Medicine, Michigan State University, East Lansing, Michigan, United States of America; University of Stellenbosch, South Africa

## Abstract

**Background:**

Only a small minority of trauma victims develops post-traumatic stress disorder (PTSD), suggesting that victims vary in their predispositions to the PTSD response to stressors. It is assumed that the role of predispositions in PTSD varies by trauma severity: when stressors are less severe, predispositions play a bigger role. In this study, we test whether the role of intelligence in PTSD varies by trauma severity. Specifically, does low intelligence plays a bigger part among victims of lower magnitude stressors than among victims of extreme stressors?

**Methods:**

Data come from a longitudinal study of randomly selected sample in Southeast Michigan (n = 713). IQ was measured at age 6. PTSD was measured at age 17, using the NIMH-DIS for DSM-IV. Stressors were classified as extreme if they involved assaultive violence (e.g. rape, sexual assault, threatened with a weapon); other stressors in the list (e.g. disaster, accidents) were classified as lower magnitude. Assaultive violence victims had experienced assaultive violence *plus* other event types or *only* assaultive violence. Victims of other stressors were participants who had never experienced assaultive violence. We compared the influence of age 6 IQ on PTSD among persons exposed to assaultive violence vs. other stressors, using multinomial logistic regression.

**Results:**

Relative risk ratio (RRR) for PTSD associated with a one point drop in age 6 IQ among victims of assaultive violence was 1.04 (95% CI 1.01, 1.06); among victims of other stressors, it was 1.03 (95% CI 0.99, 1.06). A comparison of the two RRRs indicates no significant difference between the two estimates (p = 0.652). IQ does not play a bigger role in PTSD among victims of other stressors than it does among victims of assaultive violence.

**Conclusions:**

Lower IQ exerts an adverse PTSD effect on trauma victims, with no evidence of variability by the severity of trauma they have experienced.

## Introduction

The vast majority of community residents have experienced traumatic events. Only a small minority of victims develops post-traumatic stress disorder (PTSD), suggesting that victims vary in their susceptibility to the PTSD response to traumatic experiences [1], [2], [3], [4]. Personal susceptibilities modify the probability of PTSD following traumatic experiences, enhancing or diminishing the likelihood of developing the disorder [5], [6], [7]. It has generally been assumed that the influence of predispositions is inversely related to trauma severity: exposure to extreme stressors overrides the effect of predispositions, whereas exposure to stressors of lower magnitudes allows predispositions to play a primary role [8]. Thus, the association between a predisposition and onset of PTSD should be much stronger for those who experienced low magnitude events than for those who experienced high magnitude events. Although the assumption has a compelling intuitive appeal and has been an essential part of general stress models of disease [9], until recently it has not been directly tested.

Using data from a large representative national sample, we have recently compared the PTSD effects of established predispositions – pre-existing disorders and parental psychopathology – among victims of sexual assault (a severe trauma) versus victims of each of three traumatic events of lower magnitude, accidents, disaster, and unexpected death of someone close [10]. We found that the PTSD effects of these predispositions were not significantly weaker among victims of sexual assault than among victims of less severe traumas. These predispositions predicted an elevated PTSD risk among victims of sexual assault as they did among victims of less severe events. An important predisposition not examined in that study is intelligence.

We have previously documented the role of IQ measured at age 6 in the PTSD response to subsequent trauma, based on a prospective study of children followed-up to age 17 [11]. Higher IQ protected against the PTSD response to traumatic events. Similar findings were published by others [12], [13]. Research on Vietnam veterans has also reported association between intelligence scores and the risk of PTSD [14]. A prospective study obtained pre-combat intelligence data reported that veterans with lower pre-combat intelligence were more likely to develop PTSD symptoms. The association between current intelligence and PTSD was no longer significant, after statistical adjustment for pre-combat intelligence. The authors concluded that lower pre-combat intelligence increases the risk for combat related PTSD symptoms and not that PTSD lowers intelligence [15]. A relationship between childhood IQ and a variety of later psychiatric illnesses has been reported from study of a Danish male birth cohort [16]. Previous studies on the role of IQ in PTSD did not test the hypothesis that the influence of IQ *varies* by trauma severity, specifically that it has a stronger impact when trauma is less severe. Evidence partially consistent with the hypothesis that the association of IQ with PTSD is inversely related to trauma severity – stronger when the stressor was less severe than when it was more severe – was reported by McNally and Robinaugh, based on a convenience sample of women who responded to an advertisement seeking adult survivors of child sexual abuse [17]. In that study, participants were classified according to the severity of their childhood sexual abuse, following a classification system the authors developed *ad hoc* for analysis of these data. In this study, we compare the role of IQ between two classes of traumatic events that vary markedly in their severity (pathogenicity), events involving assaultive violence and other traumatic events not involving assaultive violence. The classification of assaultive violence as extreme stressor is based on cumulative evidence that events subsumed under this rubric (e.g. rape/sexual assault, badly beaten-up, threatened with a weapon/mugged) are more pathogenic than other event types (e.g. accidents, disaster, learning of sudden death of someone close), in terms of the conditional probabilities of PTSD [10], [18]. This general finding is confirmed in this study, as reported below. Our goal is to provide a strong test of the hypothesis that the role of intelligence as predisposition for the PTSD response to trauma varies by trauma severity – stronger among victims of traumas of lesser magnitude than for traumas involving assaultive violence. We again use data from our prospective study of children followed-up from age 6, when IQ was first assessed, to age 17.

## Methods

### Ethics Statement

Written informed consent was given by parents. The Institutional Review Boards (IRBs) of the participating institutions (Henry Ford Hospital in Detroit, Michigan and Beaumont Hospital in Royal Oak, Michigan), from which the samples were drawn, and the IRB of the Michigan State University, East Lansing, Michigan, where the analysis of the de-identified data was conducted, approved the study.

### Sample and Assessment of Key Variables

The sample, study design and measurement were described in detail in previous publications [11] and are briefly summarized here. We identified and evaluated random samples of 6-year old children from the Detroit, Michigan area and re-evaluated them at age 11 and at age 17. Two major hospitals in southeast Michigan, one in the city of Detroit and the other in a middle-class suburb, were selected. In each hospital, for each year from 1983 to 1985, random samples of low birthweight and normal birthweight newborn (in equal numbers) were drawn from hospital discharge records. Of the 1095 children in the target sample, 823 (75%) participated. Of the 823 children assessed at age 6, 713 (86.6%) were assessed at age 17. The data are available upon request directed to Dr. Breslau, who is the Principal Investigator of the study.

The Wechsler Intelligence Scale for Children-Revised (WISC-R) [19] was used to measure IQ at age 6. The assessment battery included other predisposing factors, among them history of psychiatric problems. In this study we focus exclusively on IQ as a predisposition.

Lifetime PTSD was assessed at age 17 by a computerized version of NIMH-DIS for DSM-IV [20]. The assessment used a list of 14 qualifying traumatic events, following the examples given in the DSM-IV text (**Table 1**).To test the differential influence of IQ on PTSD between assaultive violence and other event types, the 14 traumatic events were classified into two categories: assaultive violence and all other event types. We classified into the assaultive violence category 1) persons who had experienced assaultive violence *plus* other event types and 2) those who had experienced *only* assaultive violence. The category of other traumatic events included persons who had never experienced assaultive violence.

**Table 1:** List of DSM-IV qualifying traumatic events.

Assaultive violence	
	Rape/sexual assault
	Held captive/tortured/kidnapped
	Shot/stabbed
	Mugged/threatened with weapon
	Badly beaten up
Other events	
	Serious accident
	Natural disaster
	Diagnosed with life-threatening illness
	Witnessed killing/serious injury
	Discovering dead body
	Break in/robbery
	Learned of trauma to others
	Learned of sudden unexpected death
	Other frightening experiences

### Statistical Analysis

We compared the influence of age 6 IQ on subsequent PTSD among persons exposed to extreme events (those involving assaultive violence) vs. its influence on PTSD among persons exposed to other events (i.e. not involving assaultive violence). We modeled PTSD and trauma type (assaultive violence vs. other event) jointly, using multinomial logistic regression. The outcome (Y) in the multinomial regression has four categories: Y = 1 if the participant experienced only non- assaultive event (never experienced assaultive violence) and did not develop PTSD; Y = 2 if the respondent experienced non-assaultive event (never experienced assaultive violence) and developed PTSD; Y = 3 if the respondent experienced assaultive violence and did not develop PTSD; and Y = 4 if the respondent experienced assaultive violence and developed PTSD. The frequency distribution of the outcome and means and standard deviations of age 6 IQ are shown in **Table 2**. In the first 4 rows of **Table 3** appear sex-adjusted relative risk ratios (RRR) for the four outcomes. The last row in the table presents the RRR of Y = 2 vs. Y = 4, which addresses the research question concerning the differential (greater) influence of age 6 IQ on PTSD following less severe trauma vs. extreme trauma (i.e. assaultive violence). Age 6 IQ was coded in negatives of the original scale so that the reported RRR indicates the effect of one point decrease in IQ on the outcome. Thus if the estimated RRR in the last row is >1.00 and if p<0.05 then the hypothesis is supported.

**Table 2:** Means and standard deviations (SD) of age-6 IQ for exposed persons classified by trauma type and presence or absence of PTSD.

	n	Mean (SD)
Other trauma/no PTSD	365	103.45 (16.64)
Other trauma/PTSD	15	96.00 (12.74)
Assaultive violence/no PTSD	131	98.51 (16.62)
Assaultive violence/PTSD	30	93.60 (13.87)

**Table 3:** Relative risk ratio (RRR) (95% CI) of PTSD due to assaultive violence vs. other trauma by age-6 IQ estimated in a multinomial regression controlling for sex.

	n	RRR (95% CI)	P-value
1. Other trauma/no PTSD	365	Reference	
2. Other trauma/PTSD	15	1.03 (0.99, 1.06)	0.090
3. Assaultive violence/no PTSD	131	1.02 (1.01, 1.03)	0.003
4. Assaultive violence/PTSD	30	1.04 (1.01, 1.06)	0.002
2. vs. 4.	–	.99 (0.95, 1.03)	0.652

Estimates 2–4 are in reference to 1(other trauma/no PTSD); 2 vs. 4 compares the two estimates of PTSD, which is the test of the hypothesis.

## Results

Of the 713 participants, 541 (75.9%) have been exposed to one or more traumatic events. Of the 541 exposed, 161 (29.8%) experienced an event involving assaultive violence. The remainder experienced other event types but never experienced assaultive violence. Of the 541 who were exposed to traumatic events, 45 (8.3%) met DSM-IV criteria for PTSD. Of the 161 who experienced assaultive violence, 30 (18.6%) developed PTSD and of the 380 who experienced events other than assaultive violence and never experienced assaultive violence, 15 (3.9%) developed PTSD. **Table 2** displays means and standard deviations (SD) of age 6 IQ across subgroups classified by type of exposure (assaultive violence vs. other event type) and the presence or absence of PTSD, a classification used in the multinomial analysis in **Table 3**. Persons who developed PTSD following either assaultive violence or other event type had lower IQ scores at age 6 than those who did not develop PTSD, according to these results. One-way ANOVA with multiple comparisons (Scheffe’s method) yielded a significant overall test (F = 6.04; df = 3; p = 0.0005), but detected no significant difference between the two PTSD groups (p = 0.975).

**Table 3** presents results from the multinomial logistic regression, estimating the effects of age 6 IQ on the PTSD risk associated with exposure to other events vs. assaultive violence. The estimates are of the relative risk ratio of the specified outcome associated with a decrease of 1 point IQ. The results show that a 1 point drop in age 6 IQ signals an increased relative risk ratio of PTSD following other trauma (not involving assaultive violence), RRR = 1.03 (95% CI, 0.99, 1.06). Similarly, a 1 point drop in age 6 IQ signals an increased PTSD relative risk ratio following assaultive violence, RRR = 1.04 (95% CI, 1.01, 1.06). A comparison of the two RRRs, presented in the last row was not significant, indicating no significant difference between the influence on PTSD of IQ between victims of non-assaultive traumas and victims of assaultive violence (p = 0.652).

Based on these results, we estimated the RRR for PTSD associated with a drop of 1 standard deviation (SD) in age 6 IQ. RRR for PTSD associated with a drop of 1 SD in IQ following other trauma (not involving assaultive violence) = 1.52 (95% CI, 0.94, 2.47) and for PTSD following assaultive violence = 1.73 (95% CI, 1.23, 2.46) (p-value is the same as in the last row of **Table 3**; not significant).

## Discussion

The question addressed in this study concerns the relationship between trauma severity and the role of predispositions in the etiology of PTSD. We tested whether the influence of IQ varies by the severity (type) of trauma the victims experienced. Does IQ exert a greater influence when trauma is less severe? We considered the subset of traumatic events involving assaultive violence (also referred to in the literature as interpersonal violence) to be extreme, judging from the frequency with which it causes PTSD, relative to other traumatic events. Our results do not support this hypothesis: the effect of IQ on the probability of PTSD did not vary between assaultive violence vs. traumatic events of lower magnitude. IQ was equally inversely related to the probability of PTSD among victims of either trauma types. A drop of one standard deviation in IQ score measured at age 6 increased the relative risk ratio of PTSD resulting from either trauma type by approximately 50%.

The results are limited by the young age – 17 years – of the participants. Peak exposure to PTSD-level events is between ages 16 and 20 years [2]. However, the conditional probability of PTSD in this study, 8.3%, falls within the range reported in surveys of adult samples in US communities. An important advantage of the study is the clear temporal order between the measurement of IQ at age 6 and the occurrence of PTSD, due to the prospective design of the study and the high follow-up completion up to age 17. As we previously reported, PTSD-level traumatic events rarely occur up to age 6, supporting the temporal priority of IQ score relative to exposure to trauma and PTSD [2], [11].D.

Our goal in this study was to test the relationship between trauma severity and the role of IQ in the etiology of PTSD. By selecting to use assaultive violence vs. other traumas not involving assaultive violence, we constructed a stark contrast of trauma severity. Future research using other categorizations of severity across trauma types would be illuminating.

The results presented here on the role of IQ in the etiology of PTSD according to trauma severity are consistent with our previous findings on other predispositions – preexisting disorders and parental psychopathology [10]. And the results of both studies – predispositions did not exert a greater effect among victims of lower magnitude stressors – correspond with an earlier meta analysis by Ozer et al (2000) that reported that the effect of several antecedent risk factors of PTSD were in fact greater (not smaller) for victims of interpersonal violence than for victims of accident, a trauma type of lower magnitude [18]. The study by McNally and Rubinaugh, which reported partial support for a greater role of IQ for victims of sexual abuse whose sexual abuse was classified as less severe, has considerable limitations, as the authors acknowledged. Chiefly, these limitations are the convenient, self-selected small sample and the *ad hoc* classification of severity of sexual abuse, a classification based on untested assumptions [17]. Although there is evidence in the literature for some of the authors’ guidelines for the classification of severity of sexual abuse (e.g., higher rates of disorders when the perpetrator had been a father than a stranger), supportive evidence is not cited. Furthermore, the assumption that closeness of relationship and repeated episodes of abuse (versus a single-episode) can be combined into a single severity index is entirely speculative. The only empirical way we know to judge severity is according to the cumulative epidemiological findings on the frequency of PTSD across trauma types or across levels of severity within types, such as Helzer reported for combat stress (wounded in combat vs. not wounded in combat) and the frequency of subsequent depression [21].

In this study, sexual abuse was included in the rape/sexual assault trauma type and classified as assaultive violence. Sexual abuse might not always involve violence. However, the absence of a separate item for sexual abuse and the low raw numbers of participants exposed to individual trauma types precludes analysis of sexual abuse in this study. Comparisons of the effect of IQ on PTSD between individual trauma types would require a far larger study.

The mechanisms through which intelligence affords protection from (or liability to) the PTSD- effects of stressors are unclear. It has been suggested that high IQ signals a general capacity to manipulate verbal information and thus a greater capacity to place traumatic experiences into meaningful concepts [22]. Lower IQ would signal a lower capacity for such cognitive processes. The contribution of our analysis is in proposing, based on our empirical results, that the influence of IQ on PTSD might apply across a wide range of traumas, in the same way that other predispositions have been observed to work [10], [18].
